# Structural Effects of pH Variation and Calcium Amount on the Microencapsulation of Glutathione in Alginate Polymers

**DOI:** 10.1155/2022/5576090

**Published:** 2022-04-13

**Authors:** Daniel Bustos, Erix W. Hernández-Rodríguez, Ricardo I. Castro, Luis Morales-Quintana

**Affiliations:** ^1^Centro de Investigación de Estudios Avanzados del Maule (CIEAM), Vicerrectoría de Investigación y Postgrado, Universidad Católica del Maule, 3460000 Talca, Chile; ^2^Laboratorio de Bioinformática y Química Computacional (LBQC), Escuela de Bioingeniería Médica, Facultad de Medicina, Universidad Católica del Maule, 3460000 Talca, Chile; ^3^Escuela de Química y Farmacia, Facultad de Medicina, Universidad Católica del Maule, 3460000 Talca, Chile; ^4^Multidisciplinary Agroindustry Research Laboratory, Instituto de Ciencias Químicas Aplicadas, Carrera de Ingeniería en Construcción, Universidad Autónoma de Chile, Talca 3467987, Chile; ^5^Multidisciplinary Agroindustry Research Laboratory, Instituto de Ciencias Biomédicas, Facultad de Ciencias de la Salud, Universidad Autónoma de Chile, Talca 3467987, Chile

## Abstract

Reduced glutathione (GSH) has a high antioxidant capacity and is present in nearly every cell in the body, playing important roles in nutrient metabolism, antioxidant defense, and regulation of cellular events. Conversely, alginate is a macromolecule that has been widely used in the food, pharmaceutical, biomedical, and textile industries due to its biocompatibility, biodegradability, nontoxicity, and nonimmunogenicity as well as for its capabilities of retaining water and stabilizing emulsions. The primary goal of this study was to characterize and optimize the formation of a molecular complex of calcium alginate with GSH using a computational approach. As methods, we evaluated the influence of varying the amount of calcium cations at two different pHs on the structural stability of Ca^2+^-alginate complexes and thus on GSH liberation from these types of nanostructures. The results showed that complex stabilization depends on pH, with the system having a lower Ca^2+^ amount that produces the major GSH release. The systems at pH 2.5 retain more molecules within the calcium-alginate complex, which release GSH more slowly when embedded in more acidic media. In conclusions, this study demonstrates the dependence of the amount of calcium and the stabilizing effect of pH on the formation and subsequent maintenance of an alginate nanostructure. The results presented in this study can help to develop better methodological frameworks in industries where the release or capture of compounds, such as GSH in this case, depends on the conditions of the alginate nanoparticle.

## 1. Introduction

Glutathione (*γ*-L-glutamyl-L-cysteinyl-glycine) is a natural tripeptide. In terms of the different glutathione forms under physiological conditions, the reduced glutathione form (GSH) is the major form and is 10- to 100-fold higher than the oxidized species oxidized GSH (GSSG) and mixed disulfide (GSSR) [1]. GSH has a high antioxidant capacity that is present in nearly every cell in the body, playing important roles in nutrient metabolism, antioxidant defense, regulation of cellular events (e.g., gene expression, protein and DNA synthesis, apoptosis, cell proliferation, and signal transduction), and detoxification of drugs and xenobiotics [2–6]. In contrast, glutathione deficiency contributes to oxidative stress and has a key role in aging and the pathogenesis of many diseases, such as seizure, Alzheimer's disease, Parkinson's disease, heart attack, cystic fibrosis, liver disease, sickle cell anemia, HIV, different cancers, stroke, and diabetes mellitus (DM) [3]. Thus, glutathione is required for several cell processes interconnected with alterations in the maintenance and regulation of the thiol-redox status due to its ability to exist in different redox species [7]. When glutathione is supplemented by dietary sources, various systemic effects have been identified, such as improvement of liver abnormalities [8–10], viral infection protection [10, 11], antitumor activity [10, 12], reduction of DM complications [10, 13], and other beneficial health effects [10].

GSH can form complexes with metals, limiting their antioxidant activity [6, 14] and moderating their ability to respond to oxidative stress [4, 6, 15]. Unfortunately, the protection that glutathione offers against oxidative decay is limited because it will quickly be lost due to oxidation reactions [16]. GSH is also sensitive to heat, light, and other environmental conditions, which may reduce its bioavailability [6, 17, 18].

One alternative to increase the stability of biologically active molecules, such as GHS, without altering their capacity for action is to use microencapsulation mediated by alginate fibers [6]. Thus, using microencapsulated calcium alginate for GSH delivery improves its bioavailability [6].

Alginate is a polysaccharide that is abundant in nature and occurs both as a structural component in marine brown algae (*Phaeophyceae*) and as a capsular polysaccharide in soil bacteria. Alginate has been widely used in the food, pharmaceutical, biomedical, and textile industries due to its biocompatibility, biodegradability, nontoxicity, and nonimmunogenicity as well as for its capabilities of retaining water and stabilizing emulsions [19–21]. The mechanical properties of alginate can be improved by mixing alginate with polyvalent metal ions, such as Ca^2+^ [22]. This process allows the binding between alginic acid and ions to produce two spatial dispositions named *β*-D-mannopyranuronate (M) and *α*-L-gulopyranuronate (G) (Figure 1(a)) [6, 23]. Thus, M and G are connected to form the alginate molecule (Figure 1(b)) [6, 23]. GSH microcapsules based on alginate polymers could offer protection against adverse environmental conditions that could compromise the antioxidant properties of this molecule and may serve as vehicles for a potentially slower or controlled release. However, in this case, GSH release depends on microcapsule stability, which is influenced by environmental factors, including the amount of calcium present. Thus, in this article, we evaluate the influence of the amount of Ca^2+^ under different acidities on the Ca^2+^-alginate complex structure, from which GSH molecules can be released as a function of the nanostructure stability.

## 2. Materials and Methods

### 2.1. Building Molecular Structures

The three-dimensional structures of *β*-D-mannopyranuronate (M) and *α*-L-gulopyranuronate (G) were sketched with MarvinSketch software v.21.8 and ChemAxon (http://www.chemaxon.com) in Linux. Then, the pKa for each subunit was evaluated with Epik [24] software from the Maestro-Schrödinger suite (L. Schrödinger Release 2021-1: Maestro, Schrödinger, “Maestro.” 2021). The pKa obtained for M ≈ 3.4 and G ≈ 3.6 (Figure 1(a)) was consistent with those reported by Chuang et al. [25]. The atomic coordinates of the GSH molecule were obtained from the cocrystallized structure of the glutathione transferase enzyme deposited in the Protein Data Bank (PDB id: 2VCV) [26, 27]. Similarly, the pKa of GSH was evaluated with Epik [24].

Only two pHs were considered in this study (2.5 and 3.6), which match the primary changes in the protonation/deprotonation effects in the M, G, and GSH subunits (Figure 1(a)). The M and G subunits were used as starting points to build two chains of alginate, involving 16 monomers in equal proportions of M and G units. One chain was built with eight consecutive subunits of G followed by eight monomers of M named G-block/M-block, while the other chain consists of eight G and M pairs named GM-block, as shown in Figure 1(b). Both chains were subjected to energy minimization in the Maestro-Schrödinger suite (Maestro, 2020) using OPLS v2005 [28] as the force field in an implicit solvent with the Polak-Ribiere Conjugate Gradient (PRCG) [29] as the minimization method with a maximum of 5000 iterations or a convergence threshold of 0.05 kcal/mol. Both alginate chains prepared previously at each pH (2.5 and 3.6) were used to generate a particle of alginate with 50 chains (25 G-block/M-block+25 GM-block) that were randomly distributed in a sphere with a 60 Å radius with PACKMOL software v.16.070.0 [30]. Correspondingly, for each system (at pH = 2.5 and 3.6), 100 GSH molecules were randomly placed in a smaller sphere with a radius of 50 Å. Finally, two calcium amounts were explored in each system using 50 and 250 Ca^2+^ ions placed in an alginate sphere with the same dimensions for all compared systems (~90.47 *μ*m^3^), as shown in Figure 1(c). Therefore, we built four different systems (I: system at pH 2.5 with 50 Ca^2+^ ions, II: system at pH 2.5 with 250 Ca^2+^ ions, III: system at pH 3.6 with 50 Ca^2+^ ions, and IV: system at pH 3.6 with 250 Ca^2+^ ions) to be simulated and analyzed in consecutive steps.

### 2.2. Molecular Dynamics Simulations

Each system was subjected to energy minimization under the same conditions as previously mentioned for monomers. Then, each system was embedded into a periodic boundary box of SPC water molecules, and an appropriate number of sodium ions were added to neutralize each system. Each system was run in the Desmond/Maestro-Schrödinger suite (Maestro, 2020) using OPLS v.2005 as the force field [28]. The default relaxation protocol was applied in five short simulations: beginning with two simulations using the NVT ensemble at low temperature, followed by three NPT simulations, the first two by 12 ps restraining the heavy atoms and one simulation by 24 ps without restraints. Finally, the simulations of production were performed in an NPT ensemble at ambient conditions (pressure = 1 atm and temperature = 300 K) with a 100 ns simulation in triplicate.

### 2.3. Postsimulation Analysis

Once the simulations were finished, we evaluated the maintenance or deformation of each particle throughout the trajectory. The radius of gyration (*R*_g_) is used as a measure of the deformation of each alginate particle during the simulation time and is defined as the root-mean-square distance of the alginate particle from its center of mass [31]. *R*_g_ was calculated with a TCL script in VMD 1.9.3 software [32]. In addition, we computed the van der Waals surface area (or molecular surface area: MSA) and the solvent-accessible surface area (SASA) of each alginate particle with the Desmond/Maestro-Schrödinger suite (Maestro, S. “Schrödinger Release 2021-1.” LLC, New York, NY, 2020, 2021). MSA and SASA are approximate measurements of the surfaces of alginate particles, and MSA is defined as the sum of the van der Waals atomic spheres that are not occluded by other atoms. SASA is calculated by rolling a spherical probe with a radius of 1.4 Å that represented a water molecule through the surface of an alginate particle. Also, we describe the deformation of alginate particles by taking conformational snapshots at the beginning, middle, and end of the simulation for the four studied configurations. To evaluate the importance of calcium ions in the maintenance of alginate particles, we count the number of calcium ions within a sphere using an *in-house* TCL script whose center is taken by the center of mass of alginate particles with a radius calculated from the *R*_g_ in every frame of the simulation. The radial distribution function (*g*(*r*)) shows that the average density of a group of atoms varies as a function of the distance from other groups of atoms and is calculated from Equation (1). In this study, *g*(*r*) and its integral were calculated to obtain the first and second coordination spheres and the coordination number. First, we measure how the G and M subunits are independently coordinated by calcium ions during the simulation time, and second, we evaluate how the calcium ions are coordinated by water molecules in each system:

(1) $$\begin{array}{c} g\left(r\right)=4\pi \;\left(\rho \left(r\right)-\rho \left(0\right)\right), \end{array}$$

where *ρ*(*r*) is the density of the atoms at a distance *r* and *ρ*(0) is the bulk density of atoms.

Both the intramolecular interactions of alginate particles and the intermolecular interactions between alginate and GSH molecules were evaluated throughout each simulation. The hydrogen bond (HB) interactions were evaluated between alginate chains and alginate-GSH using a donor-acceptor distance of 3.0 Å and an angle cutoff of ±20° from 180°. Only polar atoms were considered able to form HB using the HB plugin of VMD 1.9.3 software [32]. In addition, the salt-bridge interactions were analyzed by considering the negative partial charges of G and M and the positive partial charges of the GSH molecules with a maximum atomic distance of 3.5 Å [33]. Finally, the GSH molecules within the alginate particles were counted in a way similar to that used with calcium ions as previously described. All the data were plotted with the Gnuplot program.

## 3. Results and Discussion

To determine the capacity of the alginate polymer to encapsulate GSH under different pH conditions, we used MD simulations. Thus, we evaluated the gelation stability of calcium ions with a group of alginate chains and determined the encapsulation of GSH by the calcium-alginate complex. This analysis was based on a previous study published by the authors' laboratory that showed the capacity of the compounds to be encapsulated within the polymeric structure through noncovalent interactions [6]. We focused this study on the behavior of calcium alginate solutions at different calcium amounts and pHs. Selective and cooperative binding of calcium ions is believed to be responsible for the gelation and mechanical rigidity of alginate [34].

MD simulation studies were performed to determine whether Ca^2+^-alginate can interact in an aqueous medium under different pH conditions. First, the stability of the nanostructures containing GSH molecules was found to depend on the Ca^2+^ amount and pH when analyzing the *R*_g_, MSA, and SASA variables throughout each simulation (Figure 2). According to the MD simulations, the most stable complexes would be the two formed under conditions with a pH of 2.5, either with high or low amounts of calcium cations, as represented by the addition of 250 or 50 molecules of Ca^2+^, respectively (Figure 2(a), red and black lines). This phenomenon likely occurs because when the system is extended or relaxed, the values of the graph in Figure 2(a) increase, which also suggests that the system with the highest values tends to disassemble. This last point was verified by visual inspection of each MD simulation (Figure 3). Additionally, the molecular surface area (MSA) was evaluated, which is a measure of the nonpolar part exposed in the solvent-accessible surface area (SASA); for each system, the nonpolar zones that can form the surface of the Ca^2+^-alginate-GSH supramacromolecular system are also a way to show which is the least compressed complex. Thus, Figure 2(b) shows how the systems at pH 2.5, independent of the number of Ca^2+^, have a lower number of nonpolar regions nonoccluded (i.e., they have a lower MSA) and therefore would be less expanded or less disassembled. Finally, with respect to the surface of the different complexes, the SASA results, which is the surface with solvent access of the particle, similar to the other parameters that describe how the particle is compressed, showed that the two complexes at a pH of 2.5 have the lowest SASA, indicating that they would be more compact with respect to the two complexes at pH 3.6 (Figure 2(c)).

In particular, we observed that during the MD simulation, the GSH molecules remained encapsulated by the Ca^2+^-alginate complex when the systems were evaluated at a pH of 2.5, while the nanostructure was unstable throughout the simulation time when the pH was increased to 3.6 (Figure 3). At a pH of 2.5, both alginate monomers (M and G) are neutral, similar to GSH, which has zero total charge; therefore, this neutrality makes the particle not dependent on calcium. With respect to systems at a pH of 3.6, the G, M, and GSH molecules are negatively charged, each with a -1 charge, which makes them dependent on calcium cations (charged +2) to stabilize the complex; otherwise, the electrostatic repulsion forces the negatively charged molecules to move away from each other, as occurs in the system with a low calcium amount (Figure 3, green boxes) and to a lesser extent in the system with a pH of 3.6 but a high calcium amount (Figure 3, blue boxes).

Alginates have been increasingly used as a favorable delivery nanoplatform for biomacromolecules and a wide variety of other substances [35]. Previously, Kikuchi et al. [36] showed that high contents of G blocks of alginate can form rigid hydrogels with divalent cations such as Ca^2+^, each of which binds to two opposing G blocks in an orderly fashion, resulting in a so-called egg-box conformational arrangement. This phenomenon was similar to that described in Figure 3 but only occurs in the structures at a pH of 2.5, which is the pH that is used in most previous studies [6]. Researchers have reported that calcium ions induce chain-chain associations [6, 34–38]. Now, we have observed that this relationship exists both with calcium cations and pH (Figure 3).

Throughout the MD simulations, the pH of the medium appeared important with regard to forming and keeping the complex stable (Figure 3). However, to determine how alginate molecules behave in different environments, we analyzed the radial distribution function (RDF) of the G and M monomers. Thus, how the density of Ca^2+^ around the monomers varies was evaluated (Figure 4), allowing us to evaluate their coordination and the creation of the interaction of calcium ions crosslinking the alginate fibers in the structure called the “egg box” characteristic of calcium-alginate complexes [39]. Systems at a pH of 2.5 (Figures 4(a) and 4(b)) have a smaller RDF than systems at a pH of 3.6 (Figures 4(c) and 4(d)), suggesting that systems at a pH of 2.5 do not require coordination with calcium present, and thus, the egg-box model is unfeasible under these conditions. The results showed that the picks increased by 20 times in the case of the systems evaluated at a pH of 3.6 with respect to the two systems at a pH of 2.5. Egg boxes would also occur in these systems (at a pH of 3.6 or higher).

Now, looking at only the 3.6 pH systems (Figures 4(c) and 4(d)) and comparing them, we see that the system with a low calcium amount (e.g., only 50 calcium ions) has an RDF that is marginally higher than that with a high calcium amount (e.g., 250 ions). Particularly because the latter has more calcium ions, some calcium ions remain outside the Ca^2+^-alginate complex and therefore do not participate in the formation of egg boxes, which would affect the measurement (i.e., decreasing the RDF because it is a distance frequency). This phenomenon would not occur with the low-calcium-ion-amount system, where all the ions remain constant throughout the simulation, and all interact with alginate.

If we compare the G monomers to the M monomers, the G monomer is found to exhibit an RDF that is lower than that of the M monomer (Figures 4(c) and 4(d)). Also, and from a theoretical standpoint [39, 40], the egg-box conformation can be reached in the G monomer at a pH above its pKa (i.e., a pH of 3.6 or higher). Therefore, G monomers would coordinate the calcium ions more optimally (e.g., in the egg-box model) than M monomers due to the higher frequency identified for the latter (Figure 4(c), dark green line; Figure 4(d), dark blue line).

Figure 5 shows the integral of the RDF, which allows obtaining the number of atoms that coordinate molecules at a punctual distance [41]. In this analysis, this molecule is calcium coordinated by G or M in each system. Similar to Figure 4, in this study, the systems at a pH of 3.6 have a much higher coordination than the systems at a pH of 2.5, which again supports the fact that the latter are not coordinated by calcium. If we look only at the systems at a pH of 3.6, we see that the coordination is the same independent of the amount of calcium ions in this study; this result is correct because coordination is a physicochemical effect that is not dependent on the concentration. We also see that G and M monomers in this study have similar values; therefore, they coordinate with calcium similarly, but based on the RDF of Figure 4, there are more M monomers than G monomers around the calcium cations.

Figure 6 shows a similar analysis to that shown in Figures 4 and 5 but with water molecules around Ca^2+^ in each studied system. In Figures 6(a) and 6(b), we see that calcium ions in the systems at a pH of 2.5 have much higher RDFs and coordinations than at a pH of 3.6, which suggests that calcium is found outside of the particle on these configurations. At a pH of 2.5, the ions are retained within the particle where there are fewer coordinates by water molecules. No marked differences are found when comparing the configurations at a given pH, but differences are found at different calcium concentrations.

Finally, once we have determined the different formation parameters of the complexes at different calcium configurations under different acidity degrees corresponding to the two pHs selected according to the pKa of the molecules, we observe the interaction of this nanostructure with GSH molecules. Thus, Figure 7 shows the different interactions detected throughout the simulation between the different calcium-alginate complexes and GSH molecules. In systems at a pH of 3.6, alginate chains tend to interact more with each other than with GSH, while the opposite occurs at a pH of 2.5. These results can also be explained and corroborated by Figure 8, where the number of GSH molecules released over time is shown. The alginate particle at a pH of 3.6 has more negative charges that interact with the nitrogen that is charged positively by GSH through salt bridges that cannot exist at a pH of 2.5. Specifically, under this acidity degree, alginate is neutral, which explains the differences found for the interactions between the analyzed conditions.

Systems at a pH of 3.6 interact less with GSH because in these systems, the molecules leave the particle. In contrast, systems at a pH of 2.5 retain more GSH molecules within the particle or are released more slowly. The dependence on calcium also allows a slower (controlled) release (Figure 8, green line vs. blue line).

The analysis of complex interactions and stabilities allows for the identification of the stabilization of the polymeric structure of the Ca^2+^-alginate-GSH complex by crosslinking between the calcium ions and alginate fibers, leading to stable egg-box conformations and GSH encapsulation into the nanostructure (Figure 3). The principal complex-stabilizing forces were noncovalent interactions between functional groups in glutathione (amine, thiol, or carboxyl acid) and hydroxyl groups from the different monomers of the alginate structure. This process released more GSH molecules at a pH of 3.6 along with a small amount of calcium (Figure 8 green line), indicating that at a pH of 3.6, the amount of calcium strongly affects the GSH release rate.

## 4. Conclusion

We presented a detailed investigation of the effects of pH and the amount of calcium and the capacity to encapsulate and subsequently achieve a possible slow and controlled release of GSH molecules. Aggregate structures were shown to strongly depend on the systems at a pH of 3.6 that interact less with GHS because in these systems, the molecules leave the nanostructure formed by the complex of calcium alginate. In contrast, systems at a pH of 2.5 retained more GSH molecules within the calcium-alginate nanostructure, releasing GSH more slowly under these conditions. This study contributes to understanding the GSH release dynamics from alginate nanostructures, providing insights into the important structural effects of medium pH and calcium amount on Ca^2+^-alginate-GSH complexes that are designed to modulate the GSH release rate into a specific environment.

## Figures and Tables

**Figure 1:** Methodological scheme of the alginate particle formation: (a) pKa of *β*-D-mannopyranuronate (M), *α*-L-gulopyranuronate (G), and reduced glutathione (GSH) molecules. (b) Two blocks of alginate chains: G-block/M-block and G/M-block. (c) Alginate particle (in grayscale colors) with 100 GSH molecules (in orange color) and 50 or 250 Ca^2+^ ions (in green color).

**Figure 2:** Properties associated with the structural stability of Ca^2+^-alginate nanostructure as a function of the simulation time, under different pH conditions and Ca^2+^ amounts: (a) gyration radius (*R*_g_), (b) molecular surface area, and (c) solvent-accessible surface area.

**Figure 3:** Structural stability of Ca^2+^-alginate-GSH complexes in different pH conditions and Ca^2+^ amounts at three MD simulation times. (a) Each system at 0 ns of time; (b) each molecular system after 50 ns of MD simulation; and (c) each molecular system at the end of the MD simulation, after 100 ns. In each figure, the two blocks of alginate chains G-block/M-block and G/M-block are represented in the gray and black color, respectively, the GSH molecules are represented in orange color, and 50 or 250 Ca^2+^ ions are shown in green color.

**Figure 4:** Radial distribution function (*g*(*r*)). (a) Complex of Ca^2+^-alginate-GSH at pH 2.5 with low calcium ion amount (50 molecules); (b) complex of Ca^2+^-alginate-GSH at pH 2.5 with high calcium ion amount (250 molecules); (c) complex of Ca^2+^-alginate-GSH at pH 3.6 with low calcium ion amount (50 molecules); and (d) complex of Ca^2+^-alginate-GSH at pH 3.6 with low calcium ion amount (250 molecules).

**Figure 5:** Coordination of alginate (G and M monomers) to calcium ions. (a) Complex of Ca^2+^-alginate-GSH at pH 2.5 with low calcium ion amount (50 molecules); (b) complex of Ca^2+^-alginate-GSH at pH 2.5 with high calcium ion amount (250 molecules); (c) complex of Ca^2+^-alginate-GSH at pH 3.6 with low calcium ion amount (50 molecules); and (d) complex of Ca^2+^-alginate-GSH at pH 3.6 with low calcium ion amount (250 molecules).

**Figure 6:** (a) Radial distribution function and (b) coordination of alginate (G and M monomers) to water molecules.

**Figure 7:** Molecular interactions through simulation time: (a) Intramolecular interaction in alginate particle. (b) and (c) Hydrogen bonds and salt bridges between alginate and GSH.

**Figure 8:** Permanence of GSH molecules within the calcium-alginate nanostructure.

## Data Availability

All data are included in the manuscript.
